# An Analysis of the Cognitive Ability of Knowledge Mapping Homeschooling Based on the Rasch Model

This article has been retracted.

**DOI:** 10.1155/2022/6245984

**Published:** 2022-05-05

**Authors:** Fubao Bai, Yan Wen

**Affiliations:** School of Normal Education, Longyan University, Longyan 364012, China

## Abstract

Family cognition is a representation of the quality of family harmony, so family cognition score is an important exercise at the family level. The research based on the hybrid Rasch model is an important reference point. This study is based on the mixed Rasch model in item response theory. Firstly, descriptive statistical analysis is carried out on the family level, which is sorted according to the total score and specific proportion, and the difficulties and differences of family members in multiple choice questions at different levels are compared. Then, the number of potential categories estimated using the hybrid rush model is discussed in two cases. In one case, the number of categories is known and the categories are more detailed, so as to facilitate comparison and promote the harmony of family members.

## 1. Introduction

In the study of family function, Battick's McDermott defined family function as two categories: the overall health status or pathological status of the family. According to Mosby's Medical Dictionary [1], these two constituent conditions may be composed of multiple elements (such as cohesion, resilience, and communication skills) [2]. Early family function research is mainly aimed at different difficult groups, which is mainly used to understand and prevent dysfunctional family function and implement appropriate treatment activities when needed [3]. Over the past few decades, researchers have also created various models to evaluate family function. Among these models [4], the development of system models and evaluation tools (self-reported family questionnaire (SFI)) has been widely used in clinical and research environments [5]. Expand the SFI Research (36 questions) of [6] from a cross-cultural perspective to Chinese participants and from horizontal research design to vertical research design. Related to [7]'s five-factor model, the two-factor structure of the Chinese version of the Family Functioning Inventory (C-SFI) was confirmed to be stable and reliable across different adolescent samples in the Chinese sample and suggested that cross-cultural differences and different factor extraction techniques may be another reason for the discrepancy [8]. The two-factor structure has also been confirmed in several studies by Shek et al. In addition, C-SFI scores were significantly associated with general psychological symptoms, survival well-being, life satisfaction, and self-esteem [9], suggesting that the C-SFI could be extended to clinical psychology as an instrument for use by physicians. The lack of extension of the scale to the field of education is also a limitation of previous researchers. According to the Social Cognitive Career Development Model, the role of the family and family functioning are important moderators and mediators of family members' career planning and self-efficacy for career development (Figure 1). However, a limitation of this model is that the social component of family functioning (e.g., family health) has not been sufficiently studied in relation to family members' career-related self-efficacy. Based on the literature review, the following sections provide a critical review of research on family functioning in China, research on occupation-related variables, and research in the SEN family member population [10–12].

Family harmony focuses not only on the transfer of knowledge and skills but also on the development of cognitive ability of family members. However, the main problem with this form of score-based diagnosis is that it is impossible to explore the meaning and essence behind the test (and scores cannot be used to understand the real cognitive abilities of family members) [13–15]. For example, two family members with the same score may have different cognitive abilities and be unable to judge the difference of cognitive ability of family members with different scores. For different tests, the increase or decrease of test scores cannot indicate the change of cognitive ability of family members due to different difficulty of test papers. It can be seen that, in the era of family harmony, how to analyze the real cognitive ability of family members through examination results is a crucial proposition [16]. Based on the latent trait model Rasch model, this study designs the analysis process of family members' cognitive ability and uses the actual test results of family members to analyze their knowledge mastery and explore their real cognitive ability, so as to help the learning diagnosis from the perspective of family harmony be more scientific and accurate [17].

## 2. The Rasch Model in Education

The Rasch model is a latent trait model proposed by the Danish mathematician and statistician Georg Rasch, based on item response theory [18]. The Rasch model is an idealised mathematical model that uses a mathematical representation of individual ability, question difficulty, and the probability of an individual answering correctly [19]. The Rasch model is a probabilistic model that estimates both the difficulty of a question and the ability of a participant, where the probability of a participant answering correctly depends on the difference between the ability of the participant and the difficulty of the question [20]. When a household member's ability is equal to the difficulty of the question, the probability of getting the question right is 50%; when a household member's ability is higher than the difficulty of the question, the probability of getting the question right is higher than 50%, and the greater the difference, the greater the probability of getting the question right [21]. Similarly, when a household member's ability is lower than the difficulty of the question, the probability of getting the question right is less than 50%, and the greater the difference, the lower the probability of getting the question right. When using the Rasch model, it is better to measure when the difficulty of the question is comparable to the ability of the household members, i.e., most questions should be at the same level of difficulty as the ability of the household members, but easy questions and more difficult questions are also necessary to measure the level of all household members [22]. In general, higher difficulty questions are more appropriate for measuring high levels of household members, while lower difficulty questions have less error when measuring low levels of household members.

Fiedler et al. [23] used 150 sophomore family members at a university to analyze data from learners' final exam responses in a course using the Rasch model to propose a procedural approach that can effectively measure the reliability of a test instrument.

The study uses the Rasch model to convert family members' performance and test question difficulty into logit units and compares them on the same scale. If the mean difficulty of the test is lower than the mean performance of the family members, the test is easier; the reliability of the test is good, as reflected by the high reliability of the subjects and the reliability of the test as fitted by the Rasch model; the separation of the subjects in the set is high, reflecting the good discrimination of the test.

Outcome-based education (OBE) is a form of education that focuses on the improvement of family members' abilities and is more family-centred, with competence as the output. Under OBE, the performance of family members can be assessed through a variety of methods such as examinations, group projects, and presentations. However, it is still quite difficult to accurately measure a family member's true abilities based only on their scores in exams and projects. Field et al. [24] used the many-faceted Rasch model (MFR) to compare the effectiveness of deductive and inductive teaching. In this study, 44 extended family members were randomly divided into two groups to learn 10 grammatical structures in French class, and two different types of teaching methods were implemented.

The MFR includes more factors in the Rasch model than the ability of the family members and the difficulty of the questions, in this case, the time factor between the pre- and post-tests and the effect of the two teaching methods. Using the FACETS tool, the case was analysed separately for time-item and teaching method-item interactions, and the results showed no significant differences in question difficulty between pre- and post-tests or between groups. In the process test, by calculating the separation reliability and comparing the means of the family members' performance across the different groups, it was found that the family members showed significantly higher levels of competence than the deductive approach after receiving the inductive approach. Furthermore, residual analyses were conducted to obtain the actual performance of each family member on each topic and to understand the effectiveness of different teaching methods on different individuals [25, 26].

## 3. Hybrid Rasch Models

### 3.1. Rasch Model

According to the basic principles of the Rasch model, the probability that a particular subject will give a particular response to a particular question can be represented by a simple mathematical function consisting of the subject's ability and the difficulty of that question. The mathematical expression for this is

(1) $$\begin{array}{c} p\left(u_{ij}=1\right)=\frac{\exp\left(\theta_{j}-\beta_{i}\right)}{1+\exp\left(\theta_{j}-\beta_{i}\right)}, \end{array}$$

where *u*_*ij*_ denotes subject *j*'s score on item *i* (1 point for a correct answer, 0 points for a typo), *θ*_*j*_ denotes subject j' *s* ability, and *β*_*i*_ denotes the difficulty of item *i*.

### 3.2. Hybrid Rasch Models

The hybrid Rasch model (MRM), derived from the combination of the Rasch model and LCA [27], is one of the most widely studied and intensively used unidimensional hybrid IRT models. The expression for the probability of a correct response is

(2) $$\begin{array}{c} p\left(u_{ij}=1\right)=\sum_{c=1}^{C}\pi_{c}\times p\left(u_{ij}=1|c,\theta_{jc}\right)\\ =\sum_{c=1}^{C}\frac{\pi_{c}}{1+\exp\left(-\theta_{jc}+\beta_{ic}\right)}, \end{array}$$

where *c* denotes the potential category to which the subject belongs *c* = 1,2, ..., C, *π*_*c*_ is the size of the *c*th potential category, also called the mixing ratio, and satisfies ∑_*c*=1_^*C*^*π*_*c*_=1, *θ*_*jc*_ is the ability of subject *j* in the *c*th potential category, *βic* is the difficulty of item *i* in the *c*th potential category, and *p*(*u*_*ij*_=1*|c*, *θ*_*jc*_) is the probability that subject *j* in category *c* scores 1 on item. *i*

### 3.3. Model Selection

In this study, parameter estimation is performed for the hybrid Rasch model where the potential number of categories in the model is unknown. One approach to Bayesian estimation in a hybrid model is to treat the potential category C as an unknown parameter of a priori distribution, and in this regard, [14, 15] describe an approach in which C is an unknown parameter to be estimated. In this study, it is first assumed that the potential categorical number C is known and a particular value is taken; then, when C is unknown, different values are taken for C to obtain different models, and it is possible to choose exactly which model to use based on some theoretical basis using some appropriate statistical criteria. Model selection is a key issue in mixture modelling [28–30]. A number of previous studies have focused on the performance of the AIC criterion and the BIC criterion in determining the number of potential classes in a hybrid IRT model. These studies have consistently shown that BIC has a better chance of selecting the true number of potential classes than AIC. In this study, both the AIC and BIC criteria will be used to compare and select the optimal classification. The focus is on the performance of the AIC criterion and the BIC criterion in determining the number of potential classes in the hybrid IRT model. These studies consistently show that BIC has a better chance of selecting the true number of potential classifications than AIC. In this study, both the AIC and BIC criteria will be used to compare and select the optimal classification.

The likelihood function of the parameter to be estimated at this point is

(3) $$\begin{array}{c} L\left(\Omega \right)=\prod_{i=1}^{I}\prod_{j=1}^{J}{\left[{\left\{\sum_{c=1}^{C}\pi_{c}P\left(y_{ijc}=1|\Omega \right)\right\}}^{u_{ij}}{\left\{\sum_{c=1}^{C}\pi_{c}.\left(1-P\right)\left(y_{ijc}=1|\Omega \right)\right\}}^{1-u_{ij}}\right]}^{\sigma_{jc}^{t}}, \end{array}$$

where Ω={*c*, *θ*_*jc*_, *π*_*c*_, *β*_*ic*_}, *u*_*ij*_ denotes the score of subject *j* on item *i* (1 point for a correct answer, 0 for an incorrect answer), and *σ*_*jc*_^*t*^=1 denotes that subject *j* belongs to category *c* at step *t* of the iteration, otherwise *σ*_*jc*_^*t*^=0.

Since the value of *σ*_*jc*_^*t*^ may be different in each sample iteration, it is necessary to monitor the likelihood function at each iteration. The AIC and BIC are defined in this thesis as follows:

(4) $$\begin{array}{c} AIC=-2k^{t}+2m,\\ BIC=-2K^{t}+m*\log\;n. \end{array}$$

The model selection strategy in this study is to operate in parallel on a number of candidate models with different classifications and then accumulate information through iterations to provide a probability that a particular model can then be selected by the AIC and BIC [31].

## 4. Study Results

### 4.1. Rasch Principal Component Analysis Results

The results of the Rasch principal components' analysis showed that 43.8% of the variables in the original FH-22 and 63.2% of the variables in the short version of the FH-4 were explained by the Rasch model and that their first comparison residual eigenvalues were 2.6 and 1.7, respectively. The criteria of 2.0 (Linacre, 2020) suggest that the short version of the FH-4 meets the criteria for a unidimensional scale, whereas the unidimensional test of the original FH-22 is not supported by the data.  Table 1 presents the Rasch reliability of the original FH-22 and the short version of the FH-4 Family Health Scale. Based on the data, both versions have good item: Rasch reliability and person Rasch reliability (>0.79 for the original version and >0.80 for the short version) [12]. The item separation indices of the two versions are not very different, with the short version being slightly higher than the original. In addition, both versions have high internal consistency, with Cronbach's alpha greater than 0.85.

### 4.2. Topic Options' Setting

The option probability plots in Figure 2 reflect a single progression of the option settings (from [not at all] to [fully]) and are consistent with the underlying variables being measured. In terms of the difference in difficulty between adjacent options, the short version of the structure measure increases unidirectionally with values of −4.64, −0.87, 1.41, and 4.11 [logit], which is similar to the original version (structure measure values from −1.7, −0.7, −0.7, −0.8, −0.9, −0.9 and -0.9). −1.7, −0.89, 0.65 to 1.93) and is also in line with Linacre's (2002) recommendation of a minimum of one [logit] and a maximum of five [logits] for each level of difficulty difference in the five-level scale. This indicates that both versions function well in terms of setting options.

### 4.3. Title Rasch Model Statistical Indicators

Table 2 shows the Rasch model statistics for all items in both versions. In terms of scale fit, the short version of the FH-4 has internal and external fit values ranging from 0.8 to 1.2, with point correlation coefficients greater than 0.8, indicating that the short version items fit the Rasch model better and that all items measure the same latent variable. Most of the items in the original FH-22 fit the Rasch model well, with the exception of a few items (item 2 and item 36) where the fit exceeded 1.5; however, the point correlations for the items ranged from 0.33 to 0.80.

### 4.4. Assessment of Person Measure Invariance (PMI)

To further assess whether there are differences in measurement between the two versions, a person measure invariance plot was created based on the method provided by Bond and Fox (2015). As shown in Figure 3, the horizontal coordinate (*x*-axis) plots the [person measure] (i.e., family members' ability) measured by the original FH-22, the vertical coordinate (*y*-axis) plots the [person measure] measured by the short version of the FH-4, and the 95% control line is calculated from the person measure labeling error for each question item. As can be seen, most of the [anthropometric values] are within the error range, with the exception of a few data on the control line, indicating that there is no significant change in [anthropometric values] between the short version of the FH-4 and the original FH-22. In summary, the short version of the FH-4 maintains a high degree of internal consistency and good Rasch model reliability while streamlining redundant items and also covers a range of difficulty levels and fits the Rasch model well. In addition, the short version maintains the stability of the attributes of the human ability measure compared to the original 22-item version.

### 4.5. The Relationship between Family Health Status and Career Planning for Family Members with Special Learning Needs

Table 3 presents the performance of the career planning questions for the family members tested. The regression analysis based on the social cognitive career theory model (Figure 3) revealed that the family health variables of the family members significantly predicted the family members' career planning self-efficacy and 14.2% of the career planning self-efficacy variables could be explained by the family relationship-health variables (Figure 4). This suggests that a healthy family environment has a positive effect on the career planning development of integrated students. On another level, the promotion of career planning among integrated students can also be done from the perspective of family support by improving the family health of family members and thus enhancing their career planning development.

## 5. Conclusions

Family health profile (FH-4) has good psychometric properties. It can provide researchers in various fields with a simple screening tool to measure good family function. The study also measured the relationship between family function and career planning self-efficacy of family members with special learning needs based on the framework of social cognitive career theory. The study found that good family function (measured by family health questionnaire) is an important and positive predictor of career planning self-efficacy of family members. In view of the current situation and further research review of family function research in China, this study is the first time in China to study the relationship between family function and career planning self-efficacy in the field of inclusive education. The research results not only are a theoretical contribution to social cognitive career theory but also have an important application significance. From the perspective of family school cooperation and parents, good family function helps to improve the self-efficacy of family members' career planning.

## Figures and Tables

**Figure 1:** Social cognitive career development model.

**Figure 2:** Option probability curves.

**Figure 3:** Constant person measurements.

**Figure 4:** Pathway diagram of the relationship between family functioning, health, and career planning self-efficacy.

**Table 1:** Measurement reliability of the original FH-22 and the short version of the FH-4.

Gauge	Cronbach's alpha	Item separation index	Item Rasch reliability	Human separation index	Human Rasch reliability
FH-22	0.94	0.80	1.29	3.27	0.93
FH-4	0.85	1.99	0.81	2.38	0.86

**Table 2:** Indicator values for the topic Rasch measurements.

Scale items	Item measurement	Standard error	Internal fitness	External fitness	Point measurement correlation coefficient
Original fh-22					
fh14 R (item21)	0.41	0.12	0.98	1.01	0.66
fh13 R (item20)	0.35	0.14	1.01	1.12	0.89
fh15 R (item22)	0.37	0.12	0.67	0.65	0.78
fh16 R (item26)	0.35	0.12	1.02	0.89	0.35
fh2 R (item2)	0.33	0.12	1.5	1.87	0.35
fh10 R (item15)	0.32	0.12	0.95	0.92	0.70
fh8 R (item11)	0.21	0.12	0.85	0.85	0.66
fh7 R (item9)	0.14	0.12	0.97	0.82	0.32
fh18 R (item29)	−0.01	0.15	1.43	0.85	0.74
fh9 R (item12)	−0.08	0.15	0.73	0.74	0.89
fh4 R (item4)	−0.17	0.15	1.45	1.47	0.56
fh19 R (item33)	−0.23	0.15	0.65	0.74	0.71
fh5 R (item6)	−0.25	0.15	1.01	1.05	0.72
fh20 R (item34)	−0.31	0.15	0.72	0.69	0.75
fh3 R (item3)	−0.36	0.15	1.2	0.10	0.67
fh21 R (item35)	−0.90	0.15	0.95	0.90	0.51
Short version fh−4					
fh15R (item22)	0.70	0.20	0.99	0.95	0.83
fh1 R (item1)	0.02	0.20	0.92	0.92	0.84
fh9 R (item12)	−0.23	0.20	1.3	1.17	0.84
fh19 R (item33)	−0.50	0.20	0.87	0.83	0.87

**Table 3:** Descriptive statistics for the career planning self-efficacy questions for family members.

Scale items	Sample	Average value	Standard deviation
Career planning self-efficacy			
CP1. Be able to understand your interests and abilities well, so as to help you explore a career suitable for you	95	3.1	0.93
CP2. Can properly choose courses that are consistent with their interests and abilities to prepare for career planning	95	3.2	0.94
CP3. Can devote himself to study hard in middle school and cultivate his ability and interest in line with his post-secondary career plan	95	3.1	0.92
Career planning self-efficacy (*a* = 0.85)o	95	3.3	0.89

## Data Availability

The datasets used during the current study are available from the corresponding author upon reasonable request.
